RETRACTED

# Construct comprehensive indicators through a signal extraction approach for predicting housing price crises

**DOI:** 10.1371/journal.pone.0272213

**Published:** 2022-08-01

**Authors:** Yan Xu, Yuanting Ma, Zhengke Zhu, Jun Li, Tom Lu

**Affiliations:** 1 School of Mathematical Sciences, Ocean University of China, Qingdao, Shandong, China; 2 National Economic Engineering Laboratory, Dongbei University of Finance and Economics, Dalian, Liaoning, China; 3 School of Economics and Management, East China Jiaotong University, Nanchang, Jiangxi, China; 4 Economist of China Merchants Bank Co., LTD. Nanjing Branch, Nanjing, Jiangsu, China; 5 School of Data Science and Artificial Intelligence, Dongbei University of Finance and Economics, Dalian, Liaoning, China; 6 Department of Mathematics and Statistics, Texas Tech University, Lubbock, Texas, United States of America; University of New Mexico - Albuquerque: The University of New Mexico, UNITED STATES

## Abstract

In this paper, a novel early warning system that has usually been applied to predict the financial stress events is established to predict the likelihood of housing price crises in China. To achieve this goal, a signal extraction approach is used to monitor the evolution of a number of economic indicators that tend to exhibit the abnormal behaviors. 13 economic variables were selected as the individual indicators, and constructed as the four comprehensive indicators. Our empirical work shows that the early warning system for urban housing price crises is suitable for China’s four province-level municipalities. The in-sample forecasting results indicate the reliability of the early warning system for urban housing price crises. By studying the out-of-sample forecasting results, the likelihood of housing price crises for the four cities can be effectively predicted. We construct a novel weighted average comprehensive indicator, which performs better than the three others in terms of overall performance across all of the criteria considered in. It is shown that the extended system is more flexible in decision making than the traditional early warning system.

## 1. Introduction

In 2007, the financial tsunami triggered by the US real estate crisis quickly spread to all the corners of the globe. The US real estate market, which had been prosperous for many years, had excessively strong financial credit. Subprime mortgages were transferred and modified, which prevented the reduction or elimination of long-term systemic risks. Eventually, however, a far-reaching global financial crisis broke out. Large fluctuations in the real estate market (especially the residential market) can lead to crises in the financial industry. In particular, a crisis in the banking industry can have catastrophic consequences for a country’s entire economy. The strong economic development of the real estate industry has improved citizens’ living standards and made an undeniable contribution to the rapid growth of the national economy. However, in recent years, the housing prices of major cities in China have fluctuated violently. The meeting of the Political Bureau of the CPC Central Committee on July 24, 2017 pointed out that it is necessary to stabilize the real estate market, adhere to policy continuity and stability, and accelerate the establishment of a long-term mechanism, which put forward a policy aimed at “stabilizing the real estate market, adhering to policy continuity and stability, and accelerating the establishment of a long-term mechanism.” Therefore, an effective early warning system would be an important tool for detecting and predicting potential urban housing price crises.

RETRACTED

Most existing studies on early warning systems have focused on macroeconomic risks and financial crises, such as banking crises [1], and capital markets [2], while few studies have considered the real estate markets. [3] finds a long cycle in the real estate market. Huang and Wang [4] point out that, in order to construct an early warning system for the real estate market, it is necessary to determine early warning indicators, select early warning signals, set early warning thresholds, and classify early warning levels. [5, 6] show that three indicators can reflect the rise and fall of housing prices, including per capita income, short-term interest rate, and credit.

[7] summarize the research on currency and financial crises. They propose a signal extraction approach, also known as the KLR method, which is used to predict currency crises. The core principle is the selection of multiple early warning indicators and the determination of their early warning thresholds. When an early warning indicator reaches the corresponding critical value during a certain time period, it will issue an early warning signal. The earlier warning signals a system issues, the greater the probability that a crisis will occur in the future is. [8] considers the deficiencies in existing models for predicting the Asian financial crisis, and on the basis of individual indicators, different composite leading indicators of crises are proposed. As a result, the improved model has greatly enhanced the predictive accuracy of the KLR method.

[9] apply the KLR method to the Korean real estate market, selecting 15 individual indicators such as the interest rate, money supply, exchange rate, consumer price index (CPI), employee compensation, producer price index (PPI), new house purchases, and land supply. They use just the summed comprehensive indicator to build an early warning system for Korean real estate market crises. In addition, they define a Housing Market Pressure Index (HMPI). At each time point, they take the maximum value of the Korean housing sales price index, the Korean rental price index, the local housing sales price index, and the local rental price index to identify the possible types of Korean real estate market crises. Their research results show that the summed comprehensive indicator can accurately reflect the real estate market crises that have occurred in Korea over the years. China’s real estate market become increasing important to the national economy [10], and the operation rules of the real estate market are different from those of western countries. China’s real estate market is greatly influenced by regional policies, so an emergency index should be taken into account constructing the warning system.

RETRACTED

[11] select 12 economic indicators from the Organization of Economic Co-operation and Development (OECD), including real GDP growth rate, the exchange rate, long and short-term interest rates, the inflation rate, the housing price index, the stock market return rate, and others. They build an early warning system for financial crises by using three comprehensive indicators proposed by [8], namely, the summed comprehensive indicator, the extreme comprehensive indicator, and the weighted comprehensive indicator. They test the improved KLR model using data from 1981 to 2007, and find that these three comprehensive indicators can reflect the economic status of various countries effectively, and can send out accurate signals before a financial crisis. Although the in-sample early warning effects of the three comprehensive indicators are accurate, the test results using data from 2007Q4 to 2010Q2 show that the weighted comprehensive indicator has the best out-of-sample early warning effect on financial crises. Therefore, the authors suggest that scholars can use the weighted comprehensive indicator with the weight of the reciprocal of the noise-to-signal ratio in the early warning system for financial crises proposed by [8]. However, when the weighted comprehensive indicator is used, data with a low noise-to-signal ratio will cause a sharp increase in the weight, which in turn will lead to a sharp decline in predictive accuracy. Moreover, that situation will seriously affect the early warning accuracy of the entire model. Therefore, in this study, we reconstruct a weighted average comprehensive indicator, using “1 − *ω*^*j*^” as the weight of individual indicators. We reconstruct the fourth comprehensive indicator $CI_{t}^{4}$, which not only can reflect the early warning ability of individual indicators, but also can solve the problem of excessive weight.

RETRACTED

At present, the KLR method is mainly used for early warning research on financial and economic crises, such as crises in the currency and stock markets in China. [12] establish an early warning system for currency crises, using three test methods to investigate the degree of fit between the weighted comprehensive indicator and actual crises, these test methods include the quadratic probability score, the log probability score, and the global squared bias. However, their study remains theoretical, and those authors have not verified the effectiveness of their early warning system with empirical research. [13] conducts an empirical study, applying the KLR method to predict China’s currency crises. The author concludes that, if the early warning indicators are limited, the predicting accuracy will be affected. [14] design an economic indicator system to assess China’s economic conditions. They specifically analyze early warning signals related to China’s currency crises in recent years, and their research results show that the improved model is an effective early warning system. [15] use both the KLR method and a Probit model to build an early warning system for China’s currency market crises from 1992 to 2006. They demonstrate that the KLR method is superior to the Probit model when used to predict China’s currency crises. [16] use the KLR method to evaluate the systematic risk in China’s stock market. [17] use the KLR model to classify and study the indicators that affect the systemic risks of China’s stock market from the perspective of macro factors, micro factors, and micro factors. They obtain 9 sensitive individual indicators, and they also construct a comprehensive indicator that is weighted by the reciprocal of the noise-to-signal ratio.

Use of the KLR method to obtain early warning signals of China’s real estate market crises has just begun. [18] conducts a study based on the real estate cycle fluctuation theory and the economic early warning method, and proposes a two-dimension early warning model for the real estate market. [19] employs the KLR method, and selects six individual indicators to test their performance between 2000 and 2007. The results show that, from the perspective of house price index, China’s real estate industry had not formed a bubble. [20] uses macroeconomic variables and housing market variables from 1999Q1 to 2010Q3 to build a nationwide early warning system for China’s real estate market. The results reveal that, compared with a Probit model, the KLR model is more effective in providing early warning information about national housing crises.

RETRACTED

The literature on the KLR method in China and in other countries originally consists of a set of theoretical methods that are proposed for studying currency crises. Due to its nonparametric estimation characteristics, the KLR method can effectively avoid the shortcomings of parameter estimation methods such as model-setting errors, thus improving the predicting accuracy of the entire model. However, most scholars have applied it in the context of early warning signals for financial and economic crises such in the currency and stock markets. Less research has been conducted in terms of crises in the real estate markets. [11] discuss three comprehensive indicators (the summed comprehensive indicator, the extreme comprehensive indicator, and the weighted comprehensive indicator) in the early warning system for real estate markets in 13 OECD member countries. Most China-based studies have focused on market changes caused by real estate market cycles, and relatively few studies have addressed market changes caused by external emergencies. Furthermore, studies have not been conducted on the performance of the comprehensive indicators in China’s real estate market. China’s real estate market is characterized by large external policy shocks, such as purchase restrictions and loan restrictions. The impact of external emergencies on the real estate market is more destructive than the real estate market’s cyclical fluctuations. It is therefore of theoretical and practical significance to build an early warning system for urban housing price crises that meets China’s national conditions.

The KLR method provides a complete set of measures for building early warning indicators, early warning thresholds, monitoring ranges, and signaling horizons. Individual indicators coupled with comprehensive indicators can monitor the changes in individual economic activities and the overall macro economy at the same time. The KLR method can analyze each indicator, revealing the root of crises. The method can also predict the probability of crises. It provides a clear direction for the government to take effective measures to prevent the emergence of crises. China’s real estate market began in the 1990s and has a short development period, thus differing from the real estate markets in other countries in terms of government regulations, real estate enterprise financing and capital input allocations, as well as land factor allocations. Therefore, we cannot directly apply the early warning models for real estate market crises in other countries to predict China’s real estate market. It is necessary to select appropriate individual indicators, in order to construct comprehensive indicators that are suitable for China’s real estate market.

RETRACTED

In this paper, we propose four comprehensive indicators that may be suitable for an early warning system for China’s housing price crises, namely, the summed comprehensive indicator, the extreme comprehensive indicator, the weighted comprehensive indicator, and the weighted average comprehensive indicator. Among them, in addition to the indicators constructed by previous scholars, we also proposed an improved weighted indicator, which can overcome the problem of low accuracy of low SNR signals. By empirical analysis, we compare the performance of the four comprehensive indicators in-sample and out-of-sample. The early warning system for urban housing price crises constructed in this study can effectively identify housing price crises in China’s major cities, thereby comprehensively improving the ability to prevent systemic risks in the real estate market.

The paper is organized as follows: Section 2 provides the steps to establish the early warning system for urban housing price crises. Section 3 evaluates the performance of the four comprehensive indicators in predicting housing price crises. Section 4 provides a conclusion.

## 2. Model specification

To establish an early warning system for urban housing market crises, we need to consider the econometric model, the selection of individual indicators, the construction of comprehensive indicators, and a set of comprehensive evaluation criteria. In this paper, we adopt the KLR method to predict the probability of housing price crises within a given period of time.

### 2.1 Individual indicators

In this research, we define the signaling horizon or the forecasting horizon of a crisis, which means that economic indicators can predict the probability of crises within a specific time period. In the studies on currency crises, the signaling horizon is usually set to 24 months before a crisis. Because China’s housing system reform is no more than 20 years old, some individual indicators selected are set up for a shorter time. In this study, we set the signaling horizon at four quarters. We believe that a signal issued after four quarters is a noise signal, which does not have the predictive ability.

Let $X_{t}^{j}$ be the individual indicator j at time t, ${\overset{-}{X}}^{j}$ be the threshold of this indicator, and the binary selection variable $S_{t}^{j}$ be the signal value of the *j*th indicator at time t. If the indicator remains within its threshold boundary, it behaves normally and does not issue a signal, and thus $\;S_{t}^{j}=0$. If the indicator crosses the threshold, a signal is issued and $S_{t}^{j}=1$. That is

$$S_{t}^{j}=\left\{\begin{array}{c} 0,|X_{t}^{j}|<\left|{\bar{X}}^{j}\right|\\ 1,|X_{t}^{j}\left|\geq \right|{\bar{X}}^{j}| \end{array}\right.$$ (1)

For indicators, the threshold divides the sample interval into two areas: the normal area and the abnormal area. Obviously, there is a greater probability of a crisis in the abnormal area. If the value of an individual indicator is observed to fall in an abnormal area, then the indicator is considered to have issued an early warning signal. In order to examine the effectiveness of individual indicators, it would be useful to consider the performance of each indicator. There are four possible scenarios:

$$\begin{array}{lll} & \text{Crisis}\;\text{in}\;\text{the}\;\text{next}\;\text{four}\;\text{quarters} & \text{No}\;\text{crisis}\;\text{in}\;\text{the}\;\text{next}\;\text{four}\;\text{quarters}\\ \text{Signal}\;\text{issued} & \text{A} & \text{B}\\ \text{No}\;\text{signal}\;\text{issued} & \text{C} & \text{D} \end{array}$$

In this matrix, A is the number of quarters in which the indicator issued a correct signal, B is the number of quarters in which the indicator issued a wrong signal, C is the number of quarters in which the indicator failed to issue a signal when it should have, and D is the number of quarters in which the indicator correctly refrained from issuing a signal.

RETRACTED

Let us construct a hypothesis test. The null hypothesis is that there will be one or more crises in the next four quarters and the alternative hypothesis is that there will be no crisis in the next four quarters. Then the probability of type I errors (denoted as α) and the probability of type II errors (denoted as β) are C/(A + C) and B/(B + D). If the abnormal area is widened, the number of wrong signals will be increased and the number of missed signals will be reduced (that is, β will be increased, and α will be reduced). If the abnormal area is reduced, the number of missed signals will be increased and the number of wrong signals will be reduced (α will be increased and β will be reduced). According to mathematical statistics, α should be limited to a certain range, and β should be as small as possible. Construct ω = β/(1 –α). When α is a constant, the smaller the value of β is, the smaller the value of ω will be.

The above relationship is also the core idea in the work by [7] for determining the threshold of indicators—that is, the principle of minimum “noise-to-signal ratio”. The noise-to-signal ratio is defined as the ratio of probability that the indicator will issue a false early warning signal when there is no crisis and the probability that the indicator will issue a correct signal when there is a crisis within the next four quarters. The above ω is the noise-to-signal ratio, which is equal to [B/(B + D)]/[A/(A + C)]. [7] used the method of “grid search” method to find the optimal indicator threshold according to the principle of minimum noise-to-signal ratio. The main goal of this method is to arrange the numerical sequence of indicators in ascending order according to the size of the observed value, and to calculate the corresponding cumulative percentile (from low tail to high tail). To obtain the optimal threshold, the noise-to-signal ratio is calculated for a range of potential threshold values, and the value that minimizes the noise-to-signal ratio becomes the threshold chosen for that indicator.

RETRACTED

As we mentioned earlier, a perfect indicator should meet the ideal conditions of A > 0, B = 0, C = 0, D > 0. In such a situation, the noise-to-signal ratio of the indicator has also reached the minimum value of 0. However, it is impossible to achieve that ideal state in reality. Therefore, according to the principle of minimum noise-to-signal ratio, we construct seven criteria for screening individual indicators: the noise-to-signal ratio; the probability of crises correctly called; the conditional probability of crises given a signal; the probability of false signals with no crisis coming; the probability of crises; the probability of predicted crises in real crises; the number of predicted crises. The noise-to-signal ratio is defined as [B/(B + D)]/[A/(A + C)]. The probability of crises correctly called is defined as the percentage of the number of quarters in which a signal is followed by at least one housing price crisis within the next four quarters (A/(A + C)). The conditional probability of crises given a signal is defined as the percentage of the number of quarters in which a signal is followed by at least one housing price crisis within the next four quarters for a signal given (A/(A + B)). The probability of false signals with no crisis coming is defined as the ratio of the number of quarters in which a signal is not followed by at least one housing price crisis to the number of quarters in which no crises occur within the next four quarters (B/(B + D)). The probability of crises is defined as the percentage of the number of quarters that at least one housing price crisis occurs within the next four quarters ((A+C)/(A+B +C +D)). The probability of predicted crises in real crises is defined as the ratio of the number of quarters in which a signal is issued to the number of quarters in which at least one housing price crisis occurs within the next four quarters ((A + B)/(A + C)). The number of predicted crises is denoted as the number of quarters in which a signal is issued (A + B).

RETRACTED

It is obvious that the lower the signal-to-noise ratio is and the higher the conditional probability of crises given a signal is, the stronger the early warning capability of the indicator is. Specifically, an indicator has an early warning ability when it satisfies [B/(B + D)]/[A/(A + C)] < 1, A/(A + B) > (A + C)/(A + B + C + D).

### 2.2 Comprehensive indicators

Traditionally, it has been believed that the greater the number of signals is, the greater the probability of crises will be. This is actually an immature point of view. First of all, there are obvious differences between individual indicators, and each individual indicator has a special capability for early warning. Some forecasting results may even have conflicting results. Second, cities in different regions differ significantly from each other, and thus the potential factors that induce various cities to break out of a housing price crisis will differ. It is difficult for a single individual indicator to distinguish the differences in the housing markets between cities. Therefore, if the early warning signals issued by individual indicators can be integrated into comprehensive indicators, the amount of early warning information contained in these comprehensive indicators will be much greater than that of a single individual indicator.

During the construction of the real estate price warning model, the comprehensive indicators constructed in this paper contains much more information than a single index, and avoids the endogenous problem of multiple indexes. In addition to the indicators constructed by [11], we also propose a weighted composite indicator which is improved according to the noise signal ratio. This indicator can overcome the problem of declining accuracy caused by indicator III under the condition of low noise signal ratio, which is very important for the prediction of early warning signals.

In this paper, using the method of constructing comprehensive indicators proposed by [8], and the improved methods identified by Chinese scholars [15, 21]), we construct the following four comprehensive indicators, and compare their early warning capabilities both in-sample and out-of-sample.

#### 2.2.1 Comprehensive indicator I

Summing the value of early warning signals issued by all individual indicators at time *t*, we can obtain the first comprehensive indicator *CI*_*t*_^1^, namely the summed comprehensive indicator, which includes the early warning information of all individual indicators at time *t*.


$$CI_{t}^{1}=\overset{n}{\underset{j=1}{\sum }}S_{t}^{j}$$ (2)

RETRACTED

#### 2.2.2 Comprehensive indicator II

If $X_{t}^{j}\;>\;{\overset{-}{X}}^{j}$, an early warning signal is issued by an individual indicator. However, if the magnitude for exceeding the threshold is different, the probability of crises is also different. Obviously, an indicator with extremely aberrant behavior may predict a housing price crisis with more accuracy than one with mild behavior does. To account for this information, we define two thresholds for individual indicators: a mild threshold ${{\overset{-}{X}}_{m}}^{j}$ and an extreme threshold ${{\overset{-}{X}}_{e}}^{j}$.


$$S_{t}^{j}=\left\{\begin{array}{c} 0,\;|X_{t}^{j}|<\left|{\bar{X}}_{m}{}^{j}\right|\\ 1,\left|{\bar{X}}_{m}{}^{j}\right|\leq |X_{t}^{j}|<\left|{\bar{X}}_{e}{}^{j}\right|\\ 2,\;|X_{t}^{j}\left|\geq \right|{\bar{X}}_{e}{}^{j}| \end{array}\right.$$ (3)

Similarly, we sum the values of the mild signals and the extreme signals issued by all of the individual indicators to obtain the second comprehensive indicator, namely the extreme comprehensive indicator, which is defined as

$$CI_{t}^{2}=\overset{n}{\underset{j=1}{\sum }}\left(MS_{t}^{j}+ES_{t}^{j}\right)$$ (4)

Where ${MS}_{t}^{j}=1$ if $\left|{{\overset{-}{X}}_{m}}^{j}|\leq {|X}_{t}^{j}|<|{{\overset{-}{X}}_{e}}^{j}\right|$, $ES_{t}^{j}=2$ if ${|X}_{t}^{j}|\geq |{{\overset{-}{X}}_{e}}^{j}|$.

#### 2.2.3 Comprehensive indicator III

Comprehensive indicators I and II do not fully use the information provided by the univariate individual indicators, because neither of them accounts for the different forecasting accuracy of each individual indicator. A good way is to weight the signals of different indicators by the inverse of their noise-to-signal ratio. The third comprehensive indicator, namely the weighted comprehensive indicator, is defined as

$$CI_{t}^{3}=\overset{n}{\underset{j=1}{\sum }}\frac{S_{t}^{j}}{\omega^{j}}$$ (5)

where *ω*^*j*^ is the noise-to-signal ratio of indicator *j*.

#### 2.2.4 Comprehensive indicator IV

According to the screening criteria for individual indicators, only when the noise-to-signal ratio is less than 1 is the early warning information of individual indicators valuable. Due to the differences between individual indicators, if the inverse of each individual indicator’s noise-to-signal ratio is used to weight that indicator, the weights of the individual indicators will differ significantly. However, a too-low noise-to-signal ratio will lead to a sharp increase in the weight, which in turn will seriously affect the early warning accuracy of the entire model.

Based on the deficiency of comprehensive indicator III, we use 1 − *ω*^*j*^ as the weight of the early warning signal of individual indicators and obtain the fourth comprehensive indicator, which can not only reflect the early warning ability of individual indicators, but also solve the problem of excessive weight. The fourth comprehensive indicator, namely the weighted average comprehensive indicator, is defined as

$$CI_{t}^{4}=\overset{n}{\underset{j=1}{\sum }}\left(1-\omega^{j}\right)S_{t}^{j}$$ (6)

In theory, the fourth comprehensive indicator has the strongest early warning capability. However, in practical applications, to obtain more accurate early warning information, we use these four comprehensive indicators for comparative analysis, and we will give the best policy recommendations based on the actual forecasting results.

RETRACTED

### 2.3 Predicting housing price crises

While the comprehensive indicators contain more early warning information than the individual indicators do, we cannot infer the likelihood of the housing price crisis would happen of the city by the values. In order to obtain the probability of crises, for each value of a comprehensive indicator, we need to build an associated probability of crises within a given period of time.

For the comprehensive indicator $CI_{t}^{i},i=1,2$, the conditional probability of crises can be defined as the relative frequency of the occurrence of housing price crises within a window of h quarters when the comprehensive indicator lies in a certain interval [*ai*, *bi*).


$$P\left[C_{t,\;t+h}|CI_{t}^{i}=k\right]=\frac{Quarters\;\;with\;\;CI_{t}^{i}=k\;and\;a\;crisis\;within\;the\;next\;four\;quarters}{Quarters\;with\;CI_{t}^{i}=k}$$ (7)

For the comprehensive indicator *CI*_*t*_^*i*^, *i* = 3, 4, the conditional probability of crises can be defined as:

$$P\left[C_{t,\;t+h}|a_{i}<CI_{t}^{i}\leq b_{i}\right]=\frac{Quarters\;with\;a_{i}<CI_{t}^{i}\leq b_{i}\;\;and\;a\;crisis\;within\;\;the\;next\;four\;quarters}{Quarters\;with\;a_{i}<CI_{t}^{i}\leq b_{i}}$$ (8)

where *P* denotes probability, *C*_*t*,*t*+*h*_ is the occurrence of housing price crises in the time interval [*t*,*t* + *h*), *k* is the value of the comprehensive indicator *CI*_*t*_^*i*^,*i* = 1, 2 at time *t*, *a*_*i*_ and *b*_*i*_ denote upper and lower bound for the interval [*a*_*i*_,*b*_*i*_). The signal window is four quarters, so we set *h* = 4.

A comprehensive indicator can issue an early warning signal only when the conditional probability exceeds the critical value of the probability of crises. Here, the critical value of the probability of crises is called the “cut-off probability”. If the cut-off probability we set is too high, the number of early warning signals issued by comprehensive indicators will be too small, which will increase the probability of type I errors. If the cut-off probability is too low, the number of early warning signals issued by comprehensive indicators will be too large, which will increase the probability of type II errors. Therefore, we use the “grid search” method to find the optimal cut-off probability according to the principle of minimum noise-to-signal ratio.

RETRACTED

### 2.4 The predictive ability of comprehensive indicators

Using the conditional probability, we can employ different methods to measure the predictive ability of comprehensive indicators. [8] used an evaluation criterion called the “Quadratic Probability Score”(*QPS*) to measure the forecasting ability of comprehensive indicators. This method measures the average difference between the probability of the occurrence of an actual housing price crisis (represented by a dummy variable *R*_*t*_) and the probability of a predicted housing price crisis (represented by *P*_*t*_). Here, *P*_*t*_ is the conditional probability of crises given a signal. The calculation formula of the *QPS* is

$$QPS^{j}=\frac{1}{T}\overset{T}{\underset{t=1}{\sum }}2{\left(P_{t}^{j}-R_{t}\right)}^{2}$$ (9)

where *QPS*^*j*^ represents the quadratic probability score of the comprehensive indicator *CI*_*t*_^*j*^, and *T* represents the time of the entire sample. Obviously, the range of the *QPS* values is between the interval [0, 2]. A value of *QPS* = 0 means that the comprehensive indicator has complete early warning capability, and *QPS* = 2 means that the comprehensive indicator has no early warning capability. In other words, the smaller the *QPS* value is, the stronger the forecasting ability of the comprehensive indicator is.

In addition, the forecasting evaluation is based on five different criteria: the noise-to-signal ratio; the probability of crises correctly called; the conditional probability of crises given a signal; the probability of safety correctly predicted; the conditional probability of crises given no signal. The noise-to-signal ratio is defined as [*B/*(*B* + *D*)]*/*[*A/*(*A* + *C*)]. The probability of crises correctly called is defined as the percentage of the number of quarters in which a signal is followed by at least one housing price crisis within the next four quarters (*A/*(*A* + *C*)). The conditional probability of crises given a signal is defined as the percentage of the number of quarters in which a signal is followed by at least one housing price crisis within the next four quarters for given a signal (*A/*(*A* + *B*)). The probability of safety correctly predicted is defined as the percentage of the number of quarters in which a signal is not issued and housing price crises will not happen within the next four quarters (*D/*(*B* + *D*)). The conditional probability of crises given no signal is defined as the percentage of the number of quarters in which a signal is not issued, but at least one housing price crisis occurs within the next four quarters (*C/*(*C* + *D*)).

RETRACTED

In an ideal situation, a perfect comprehensive indicator should meet the following conditions: *QPS* = 0, *B/*(*B* + *D*)]*/*[*A/*(*A* + *C*) = 0,*A/*(*A* + *C*) = 1,*D/*(*B* + *D*) = 1,*A/*(*A* + *B*) = 1,*C/*(*C* + *D*) = 0.

## 3. An empirical analysis

Because of the availability of the data, we select Beijing, Shanghai, Tianjin, and Chongqing as the research objects. The time span is from 2005Q3 to 2018Q4. Data are obtained from the China Economic Network Statistics Database, China Economic Network Industry Database, Wind Information, and the National Bureau of Statistics. On the basis of existing studies on the real estate market in China, we select 13 economic variables as individual indicators. These include the M2 growth rate, the exchange rate, the SSE Real Estate, the inflation rate, the medium-term and long-term loan interest rates, the ratio of the completed residential investment in real estate enterprises to the completed residential investment in fixed assets, the ratio of residential property sales to the GDP, the ratio of residential area for sales to the completed residential area, the ratio of residential area under construction to the completed residential area, the residential CPI, the funds in place for real estate enterprises, the land transaction price for real estate enterprises, and the GDP growth rate. Among the 13 variables, the Sse Real Estate index is a real-time reflection of the sudden situation of the real estate market, as well as the most real response of real estate prices driven by policy factors, which is exactly the signal of reginal policies. We integrate the early warning information from those individual indicators into four comprehensive indicators. The reliability of the early warning system for crises in the urban housing market is verified through the in-sample early warning results. In addition, current housing price movements in the four urban housing markets are analyzed through the out-of-sample results and the crisis prediction probability curves.

China is not a complete market economy, and regional real estate price control policies have a significant impact on the real estate market, which differs from city to city, which are complex and difficult to simulate, and when real data are available, it is often better to choose real statistics. Because some of the selected individual indicators have both monthly and quarterly data, some individual indicators only have monthly data, and others only have quarterly data, we use quarterly data only in order to ensure the accuracy and reliability of the data. For individual indicators with only monthly data, we adopt the price index conversion method with a fixed base. We first convert monthly chain data to monthly fixed data (with the base period being December 2005), then convert the monthly fixed data to quarterly fixed data (with the base period being 2005Q4), and finally we calculate quarterly year-on-year data. Because the absolute value of the indicator variable is relatively large, in order to facilitate comparison, we convert all indicator variables into relative values of year-on-year or comparison with other variables.

RETRACTED

We take the first three policy cycle time periods of China’s real estate market (from 2005Q3 to 2014Q2) as the in-sample time for building an early warning system for urban housing price crises in China. We use the fourth policy cycle time period (from 2014Q3 to 2018Q4) to evaluate the out-of-sample performance of the early warning system for urban housing price crises.

### 3.1 Urban housing price crises

In this paper, we use the method by [11] to identify financial crises, and we define the housing price crises of the four major cities we choose in China as follows:

$$hps_{t}=\left\{\begin{array}{c} 1,\;r_{t}>\mu_{r}+k\sigma_{r}\\ 0,\;\;\;\;\;\;otherwise \end{array}\right.$$ (10)

The dummy variable *hps*_*t*_ reflects the housing market risk at time *t*, *r*_*t*_ is the housing price index at time *t* (using the larger value between the new housing sales price index and the second-hand housing sales price index over the same period as the current housing price index), *μ*_*r*_ and *σ*_*r*_ are the sample mean and standard deviation, respectively, of the housing price index, *k* is the threshold coefficient, and *μ*_*r*_ + *kσ*_*r*_ is called the threshold of a housing price crisis.

Once the residential price index at time *t* exceeds the threshold (*r*_*t*_ *> μ*_*r*_ + *kσ*_*r*_), indicating that the residential price growth rate is too fast during a period, the housing market shows risk of “overheating” (*hps*_*t*_ = 1), and the government needs to take appropriate regulatory measures to slow down the residential price growth rate and to”cool down” the local residential market.

The coefficient *k* plays a very important role in determining the threshold of the housing price crisis in Eq 10. By consulting the relevant historical literature, we find that studies in China and abroad have not yet developed a theoretical method for effectively determining the coefficient *k*. Thus, we use empirical methods to find the appropriate threshold for coefficient *k*. In the extant research on early warning systems for financial crises, the threshold coefficient *k* mainly has the following values: [22] take *k* = 2; [23] take *k* = 1; [11] take *k* = 1.5.

RETRACTED

Fig 1 displays the housing price crisis trend for Beijing, Shanghai, Tianjin, and Chongqing when the threshold coefficient *k* = 1, 1.5, and 2. The housing price crisis identified by *k* = 1 is generally consistent with the policy cycle of China’s real estate market. After comparative empirical analysis, when *k* = 1, we obtain the most accurate predictions for the housing price crises. Therefore, we select *k* = 1 as the threshold coefficient.

**Fig 1:** Housing price indexes for selected cities. The solid lines are the growth rates of housing prices. The dashed lines are crisis-identification thresholds with k = 1, 1.5 and 2.

Fig 1 indicates some interesting results. First, the housing price indexes for Beijing and Shanghai break through the critical value at the end of 2015, and they begin to fall after reaching their highest values in 2016. At the end of 2018, the housing prices in Beijing and Shanghai stabilize at a low level. This indicates that a series of regulatory measures that are implemented by the government have worked very well. At the same time, it can be observed that Beijing’s housing price has rebounded in early 2019, but it is still below the threshold. Second, Tianjin’s housing price index quickly breaks through the threshold after reaching its highest point in mid-2016. It then falls back to a lower level below the threshold during 2018, thus indicating that the 331 New Deal implemented by the government has stabilized Tianjin’s housing prices and kept them low (On March 31, 2017, the Tianjin Municipal People’s Government published the Implementation Opinions of the General Office of Tianjin Municipal People’s Government on Further Deepening the Regulation and Control of the Real Estate Market in Tianjin. The opinions pointed out that households with local registration are restricted to purchase the third set, and households with non-local registration are restricted to purchase the second set.). However, Tianjin’s housing prices begin to rise again in early 2019. This may have been due to the implementation of the Tianjin Settlement Policy in 2018 (In May 2018, Tianjin Municipal People’s Government promulgated the “Implementation Measures for the Introduction of Talents in Tianjin”.). Third, Chongqing’s housing price index has been on an upward trend in recent years. It breaks through the threshold in 2017, but in 2018 it falls temporarily. This indicates that a series of regulatory policies implemented by the Chongqing government has achieved a certain effect (On June 28, 2018, Chongqing issued the”Notice on Further Strengthening the Regulation of the Real Estate Market”. According to the requirements of the”Notice”, Chongqing will further strengthen the regulation of the real estate market considering the current market situation). However, we can see that the price index for Chongqing has gradually recovered and then it breaks through the threshold in early 2019, creating a housing price crisis.

RETRACTED

### 3.2 Selection of individual indicators

Based on existing studies related to China’s real estate early warning system, 13 individual indicators are initially selected from the national and local levels, as shown in Table 1.

**Table 1:** Interpretation of individual indicators.

Category	Indicator	Rename
National level	Growth rate of M2	Indicator 1
	Exchange rate	Indicator 2
	SSE Real Estate	Indicator 3
	Inflation rate	Indicator 4
	Interest rates of medium-term and long-term loan	Indicator 5
Local level	Ratio of the completed residential investment in real estate enterprises to the completed residential investment in fixed assets	Indicator 6
	Ratio of the residential sales to the GDP	Indicator 7
	Ratio of the residential area for sales to the completed residential area	Indicator 8
	Ratio of the residential area under construction to the completed residential area	Indicator 9
	Residential CPI	Indicator 10
	Funds in place for real estate enterprises	Indicator 11
	Land transaction price for real enterprises	Indicator 12
	Growth rate of GDP	Indicator 13

Note: This table presents 13 individual indicators selected from both national and local levels.

For this paper, we use historical data on the four cities to process the selected individual indicators under low tail (10% -30%) conditions and high tail (70% -90%) conditions simultaneously. We select the optimal threshold of individual indicators based on the minimum noise-to-signal ratio. The results are shown in Table 2.

**Table 2:** Performance of the individual indicators in the KLR tests.

Indicator	Threshold percentile	$\frac{A}{A+C}$	$\frac{B}{B+D}$	Noise/signal ratio	$\frac{A}{A+B}$	$\frac{A+C}{A+B+C+D}$	$\frac{A+B}{A+C}$	A+B
Indicator 1(L)	23	0.15	0.31	2.16	0.22	0.38	0.20	5
**Indicator 1(H)**	**86**	**0.36**	**0.00**	**0.03**	**1.00**	**0.38**	**0.44**	**11**
Indicator 2(L)	14.5	0.13	0.19	1.50	0.29	0.38	0.20	5
**Indicator 2(H)**	**89**	**0.15**	**0.09**	**0.62**	**0.50**	**0.38**	**0.16**	**4**
Indicator 3(L)	11.5	0.13	0.15	1.15	0.35	0.38	0.52	13
**Indicator 3(H)**	**77.5**	**0.40**	**0.11**	**0.28**	**0.69**	**0.38**	**0.72**	**18**
**Indicator 4(L)**	**10.5**	**0.25**	**0.02**	**0.09**	**0.88**	**0.38**	**0.52**	**13**
Indicator 4(H)	86	0.11	0.16	1.44	0.30	0.38	0.20	5
**Indicator 5(L)**	**10**	**0.42**	**0.06**	**0.13**	**0.82**	**0.38**	**0.44**	**11**
Indicator 5(H)	83	0.15	0.18	1.24	0.33	0.38	0.20	5
Indicator 6(L)	18	0.13	0.21	1.68	0.27	0.38	0.40	10
**Indicator 6(H)**	**72**	**0.36**	**0.22**	**0.62**	**0.50**	**0.38**	**0.48**	**12**
Indicator 7(L)	26.5	0.07	0.38	5.25	0.11	0.38	0.16	4
**Indicator 7(H)**	**90**	**0.18**	**0.04**	**0.25**	**0.71**	**0.38**	**0.56**	**14**
Indicator 8(L)	14.5	0.13	0.16	1.24	0.33	0.38	0.52	13
**Indicator 8(H)**	**90**	**0.16**	**0.06**	**0.34**	**0.64**	**0.38**	**0.64**	**16**
Indicator 9(L)	11	0.16	0.08	0.48	0.56	0.38	0.60	15
**Indicator 9(H)**	**72**	**0.33**	**0.25**	**0.76**	**0.45**	**0.38**	**1.00**	**25**
**Indicator 10(L)**	**10.5**	**0.25**	**0.01**	**0.04**	**0.93**	**0.38**	**0.44**	**11**
Indicator 10(H)	90	0.09	0.10	1.11	0.36	0.38	0.12	3
Indicator 11(L)	13	0.09	0.16	1.73	0.26	0.38	0.28	7
**Indicator 11(H)**	**90**	**0.25**	**0.00**	**0.04**	**1.00**	**0.38**	**0.60**	**15**
**Indicator 12(L)**	**10.5**	**0.16**	**0.07**	**0.41**	**0.60**	**0.38**	**0.64**	**16**
Indicator 12(H)	76.5	0.22	0.25	1.13	0.35	0.38	0.76	19
Indicator 13(L)	17.5	0.29	0.10	0.35	0.64	0.38	0.36	9
**Indicator 13(H)**	**73**	**0.29**	**0.25**	**0.85**	**0.42**	**0.38**	**0.60**	**15**

Note: The estimation period is from 2005Q3 to 2017Q2 using data from Beijing, Shanghai, Tianjin, and Chongqing. The threshold percentile, which minimizes the noise-to-signal ratio, is obtained by using a grid search over the risk tail and is used to determine the optimal threshold. The noise-to-signal ratio is defined as the ratio of false signals *B/*(*B* + *D*) to good signals *A/*(*A* + *C*).

RETRACTED

Using the screening criteria of individual indicators in section 2.1, we first select the indicators with a noise-to-signal ratio that is less than 1 under low-tail and high-tail conditions: indicator 1 (H), indicator 2 (H), indicator 3 (H), indicator 4 (L), indicator 5 (L), indicator 6 (H), indicator 7 (H), indicator 8 (H), indicator 9 (L), indicator 9 (H), indicator 10 (L), indicator 11 (H), Indicator 12 (L), indicator 13 (L), and indicator 13(H). Among them, the noise-to-signal ratios of indicators 9 and 13 under low-tail and high-tail conditions are less than 1. However, indicator 9(H) performs better in terms of its ability to correctly call crises, and indicator 13(H) has a larger number of predicted crises, so we select indicator 9(H) and indicator 13(H) for further study.

Table 2 shows that the noise-to-signal ratios of indicator 1 (H), indicator 4 (L), indicator 10 (L), and indicator 11 (H) are much lower than 1, indicating that these four indicators have extremely strong early warning capabilities. When policy makers formulate real estate policies, therefore, they should focus on monitoring the changes in these four indicators. In summary, the individual indicators we select are as follows: indicator 1 (H), indicator 2 (H), indicator 3 (H), indicator 4 (L), indicator 5 (L), indicator 6 (H), indicator 7 (H), indicator 8 (H), indicator 9 (H), indicator 10 (L), indicator 11 (H), indicator 12 (L), and indicator 13 (H).

RETRACTED

We use historical data from four cities in China, and calculate the conditional probability of crises given a signal and the cut-off probabilities of the comprehensive indicators, as shown in Tables 3 and 4.

**Table 3:** Conditional probabilities of crises given a signal associated with comprehensive indicators.

Comprehensive Indicator I		Comprehensive Indicator II		Comprehensive Indicator III		Comprehensive Indicator IV	
Value	Probability	Value	Probability	Value	Probability	Value	Probability
1	0.241	1	0.241	(0,15.2]	0.257	(0,0.95]	0.209
2	0.205	2	0.179	(15.2,30.5]	0.444	(0.95,1.91]	0.333
3	0.125	3	0.158	*>* 30.5	1.000	(1.91,2.87]	0.889
4	0.435	4	0.333	(45.8,61.1]	1.000	*>* 2.87	1.000
5	0.800	5	0.231				
*>* 6	1.000	6	0.636				
		*>* 7	1.000				

Note: This table shows the conditional probabilities of crises given a signal for comprehensive indicator I through IV. The probabilities are calculated by Eqs (7) and (8).

**Table 4:** Cut-off probabilities.

Comprehensive Indicator I		Comprehensive Indicator II		Comprehensive Indicator III		Comprehensive Indicator IV	
Threshold	Noise/signal ratio	Threshold	Noise/signal ratio	Threshold	Noise/signal ratio	Threshold	Noise/signal ratio
0.20	0.81	0.20	0.66	0.20	1.00	0.20	1.00
0.25	0.25	0.25	0.30	0.25	1.00	0.25	0.29
0.30	0.25	0.30	0.30	0.30	0.12	0.30	0.29
0.35	0.25	**0.35**	**0.08**	0.35	0.12	**0.35**	**0.02**
0.40	0.25	0.40	0.08	0.40	0.12	0.40	0.02
**0.45**	**0.05**	0.45	0.08	**0.45**	**0.00**	0.45	0.02
0.50	0.05	0.50	0.08	0.50	0.00	0.50	0.02

Note: This table shows the cut-off probabilities we selected for comprehensive indicator I through IV. The cut-off probability for each comprehensive indicator comes from the in-sample estimation by minimizing the noise-to-signal ratio.

Table 3 shows that the conditional probability of crises given a signal increases as the value of the comprehensive indicator increases. It can be seen from Table 4 that, according to the principle of minimum noise-to-signal ratio, the cut-off probabilities of the four comprehensive indicators are 0.45, 0.35, 0.45, and 0.35. Once the conditional probability of crises given a signal exceeds the cut-off probability, the early warning system will issue a signal, and the government needs to take measures to prevent housing prices from rising too fast.

RETRACTED

### 3.3 Performance of the comprehensive indicators

Table 5 shows the in-sample and out-of-sample forecasting results of the four comprehensive indicators in the early warning system for Beijing’s housing price crises.

**Table 5:** Predictive ability from the comprehensive indicators.

**In-sample** 2005Q3-2014Q2	**Beijing**			
Comprehensive indicator	I	II	III	IV
Cut-off probability	0.45	0.35	0.30	0.35
Quadratic Probability Score	0.37	0.33	0.40	0.36
Noise-to-signal ratio	0.11	0.00	0.00	0.00
Probability of crises correctly called	0.44	0.50	0.38	0.44
Probability of safety correctly predicted	0.95	1.00	1.00	1.00
Conditional probability of crises given a signal	0.88	1.00	1.00	1.00
Conditional probability of crises given no signal	0.32	0.29	0.33	0.31
**Out-of-sample** 2014Q3-2018Q4 Quadratic Probability Score	0.70	0.81	0.67	0.70
Noise-to-signal ratio	NaN	Inf	NaN	NaN
Probability of crises correctly called	0.00	0.00	0.00	0.00
Probability of safety correctly predicted	1.00	0.91	1.00	1.00
Conditional probability of crises given a signal	NaN	0.00	NaN	NaN
Conditional probability of crises given no signal	0.50	0.52	0.50	0.50

Note: The cut-off probability for each comprehensive indicator comes from the in-sample estimation by minimizing the noise-to-signal ratio. The probability of crises correctly called is defined as *A/*(*A* + *C*); the probability of safety correctly predicted is defined as *D/*(*B* + *D*); the conditional probability of crises given a signal is defined as *A/*(*A* + *B*); the conditional probability of crises given no signal is defined as *C/*(*C* + *D*). “NaN”, standing for not a number, is a numeric data type value representing an undefined or unrepresentable value. “Inf”, standing for infinity, describes something without any bound or larger than any number.

The in-sample results from Beijing reveal some interesting findings. First, the *QPS* and noise-to-signal ratios of the four comprehensive indicators are less than 1, indicating that these indicators are useful tools for predicting housing price crises. Second, comprehensive indicator IV performs better than or equal to both comprehensive indicator I and III in terms of its ability to correctly call housing price crises, to correctly predict non-housing price crises, to predict housing price crises given a signal, and to predict housing price crises given no signal. Furthermore, comprehensive indicator II performs better than comprehensive indicator IV in terms of its ability to correctly call housing price crises and to predict housing price crises given no signal. One explanation for this result is that although the summed comprehensive indicator contains aggregate information, it does not account for the different forecasting accuracy of each individual indicator. For the weighted comprehensive indicator, a too-low noise-to-signal ratio will lead to a sharp increase in the weight, which will seriously affect the forecasting accuracy. In contrast, the weighted average comprehensive indicator puts more weight on the signals issued by indicators and avoids the problem of excessive weight. Therefore, it is reasonable that comprehensive indicators II and IV would perform better than the other comprehensive indicators across all the criteria considered.

RETRACTED

In summary, the in-sample results from Beijing suggest that the four comprehensive indicators are informative for predicting housing price crises. Specifically, comprehensive indicators II and IV have a better performance than the other two comprehensive indicators do, across all the criteria considered.

The out-of-sample results from Beijing reflect the out-of-sample forecasting accuracy of the four comprehensive indicators. The *QPS* values of the four comprehensive indicators are less than 1, indicating that these indicators are useful tools for predicting housing price crises. In contrast, comprehensive indicator II performs poorly in terms of its ability to correctly predict non-housing price crises and to predict housing price crises given no signal. However, for most of the comprehensive indicators, both the numerator and the denominator of the noise-to-signal ratio are zero in the out-of-sample forecasting results. Therefore, it is not easy to examine comprehensively the out-of-sample prediction ability of the four comprehensive indicators.

Fig 2. plots the forecasted probabilities of housing price crises for the four comprehensive indicators (*k* = 1). It is obvious that some comprehensive indicators have captured the abnormal situation before a crisis. First, comprehensive indicator I repeatedly jumps and fluctuates outside the sample. It has risen significantly to reach the cut-off probability in 2015 and 2017, and it weakly predicts the housing price crisis that occurred in 2015 and 2017. However, it failed to predict the housing price crisis that occurred in 2016. Second, comprehensive indicator II rises and almost reaches the cut-off probability during 2016, weakly predicting the housing price crisis that occurred in that year. Third, comprehensive indicator IV remains at a stable level far below the cut-off probability after 2011. Then it has risen sharply after 2014, mostly fluctuating around the cut-off probability. Finally, comprehensive indicator III performs poorly, remaining at a stable level far below the cut-off probability after 2011.

RETRACTED

**Fig 2:** Probability forecasts of housing price crises for Beijing. The shaded regions represent the time spans of housing price crises. The solid lines are the forecasted probabilities from the four comprehensive indicators with the threshold level of *k* = 1. Correspondingly, the dashed lines are their cut-off probabilities.

Table 6 shows the in-sample and out-of-sample forecasting results of the four comprehensive indicators in the early warning system for Shanghai’s housing price crises.

**Table 6:** Predictive ability from the comprehensive indicators.

**In-sample** 2005Q3-2014Q2	**Shanghai**			
Comprehensive indicator	I	II	III	IV
Cut-off probability	0.45	0.35	0.45	0.35
Quadratic Probability Score	0.43	0.40	0.44	0.43
Noise-to-signal ratio	0.13	0.13	0.00	0.13
Probability of crises correctly called	0.41	0.41	0.29	0.41
Probability of safety correctly predicted	0.95	0.95	1.00	0.95
Conditional probability of crises given a signal	0.88	0.88	1.00	0.88
Conditional probability of crises given no signal	0.36	0.36	0.39	0.36
**Out-of-sample** 2014Q3-2018Q4 Quadratic Probability Score	0.69	0.80	0.67	0.67
Noise-to-signal ratio	NaN	NaN	NaN	NaN
Probability of crises correctly called	0.00	0.00	0.00	0.00
Probability of safety correctly predicted	1.00	1.00	1.00	1.00
Conditional probability of crises given a signal	NaN	NaN	NaN	NaN
Conditional probability of crises given no signal	0.55	0.55	0.55	0.55

Note: The cut-off probability for each comprehensive indicator comes from the in-sample estimation by minimizing the noise-to-signal ratio. The probability of crises correctly called is defined as *A/*(*A* + *C*); the probability of safety correctly predicted is defined as *D/*(*B* + *D*); the conditional probability of crises given a signal is defined as *A/*(*A* + *B*); the conditional probability of crises given no signal is defined as *C/*(*C* + *D*).”NaN”, standing for not a number, is a numeric data type value representing an undefined or unrepresentable value.

The in-sample results from Shanghai offer some interesting findings. First, the *QPS* and noise-to-signal ratios of the four comprehensive indicators are less than 1, indicating that these indicators are useful tools for predicting housing price crises. Second, comprehensive indicator IV performs equal to both comprehensive indicators I and II in terms of its ability to correctly call housing price crises, to correctly predict non-housing price crises, to predict housing price crises given a signal, and to predict housing price crises given no signal. Furthermore, comprehensive indicator IV performs better than comprehensive indicator III in terms of its ability to correctly call housing price crises, and to predict housing price crises given no signal. One explanation for this result is that although the summed comprehensive indicator and the extreme comprehensive indicator contain aggregate information, they cannot account for the different forecasting accuracy of each indicator. For the weighted comprehensive indicator, a too-low noise-to-signal ratio will lead to a sharp increase in the weight, which in turn will seriously affect the forecasting accuracy. In contrast, the weighted average comprehensive indicator puts more weight on the signals issued by indicators and avoids the problem of excessive weight. Therefore, it is reasonable that comprehensive indicator IV performs better at both correctly calling housing price crises and at predicting housing price crises given no signal.

RETRACTED

In summary, the in-sample results from Shanghai suggest that the four comprehensive indicators are informative for predicting housing price crises. Specifically, comprehensive indicator IV has a better performance than comprehensive indicator III does, in terms of its ability to correctly call housing price crises, and to predict housing price crises given no signal.

The out-of-sample results from Shanghai reflect the out-of-sample forecasting accuracy of the four comprehensive indicators. The *QPS* values of the four comprehensive indicators are less than 1, indicating that these indicators are useful tools for predicting housing price crises. The four comprehensive indicators have the same performance in terms of their ability to correctly predict non-housing price crises and to predict housing price crises given no signal. However, for the four comprehensive indicators, both the numerator and the denominator of the noise-to-signal ratio are zero in the out-of-sample forecasting results. Therefore, it is difficult to examine comprehensively the out-of-sample prediction ability of the four comprehensive indicators.

Fig 3 plots the forecasted probabilities of housing price crises for the four comprehensive indicators (*k* = 1). It is obvious that some comprehensive indicators capture the abnormal situation before a crisis. First, comprehensive indicator I repeatedly jumps and fluctuates outside the sample. The highest point of each fluctuation is close to the cut-off probability, which weakly predict Shanghai’s housing price crises that occurred in 2016 and 2017. Second, comprehensive indicator II rises to near the cut-off probability in 2016 and 2017. Third, comprehensive indicator IV has repeatedly jumped and fluctuated from 2015 on to reach the cut-off probability. By comparison, comprehensive indicator III performs poorly, remaining at a stable level far below the cut-off probability after 2014.

RETRACTED

**Fig 3:** Probability forecasts of housing price crises for Shanghai. The shaded regions represent the time spans of housing price crises. The solid lines are the forecasted probabilities from the four comprehensive indicators with the threshold level of *k* = 1. Correspondingly, the dashed lines are their cut-off probabilities.

Table 7 shows the in-sample and out-of-sample forecasting results of the four comprehensive indicators in the early warning system for Tianjin’s housing price crises.

**Table 7:** Predictive ability from the comprehensive indicators.

**In-sample** 2005Q3-2014Q2	**Tianjin**			
Comprehensive indicator	I	II	III	IV
Cut-off probability	0.45	0.35	0.45	0.35
Quadratic Probability Score	0.18	0.21	0.24	0.17
Noise-to-signal ratio	0.00	0.10	0.00	0.00
Probability of crises correctly called	0.60	0.80	0.50	0.70
Probability of safety correctly predicted	1.00	0.92	1.00	1.00
Conditional probability of crises given a signal	1.00	0.80	1.00	1.00
Conditional probability of crises given no signal	0.13	0.08	0.16	0.10
**Out-of-sample** 2014Q3-2018Q4 Quadratic Probability Score	0.58	0.52	0.48	0.49
Noise-to-signal ratio	0.57	0.43	0.00	0.29
Probability of crises correctly called	0.13	0.50	0.13	0.25
Probability of safety correctly predicted	0.93	0.79	1.00	0.93
Conditional probability of crises given a signal	0.50	0.57	1.00	0.67
Conditional probability of crises given no signal	0.35	0.27	0.33	0.32

Note: The cut-off probability for each comprehensive indicator comes from the in-sample estimation by minimizing the noise-to-signal ratio. The probability of crises correctly called is defined as *A/*(*A* + *C*); the probability of safety correctly predicted is defined as *D/*(*B* + *D*); the conditional probability of crises given a signal is defined as *A/*(*A* + *B*); the conditional probability of crises given no signal is defined as *C/*(*C* + *D*).

The in-sample results from Tianjin also reveal some interesting findings. First, the *QPS* values and noise-to-signal ratios of the four comprehensive indicators are less than 1, indicating that these indicators are useful tools for predicting housing price crises.

Second, comprehensive indicator IV performs better than both comprehensive indicators I and III in terms of its ability to correctly call housing price crises and to predict housing price crises given no signal. Third, comprehensive indicator IV performs better than comprehensive indicator II in terms of its ability to correctly predict non-housing price crises and to predict housing price crises given a signal. One explanation for this result is that while the summed comprehensive indicator and the extreme comprehensive indicator contain aggregate information, they cannot account for the different forecasting accuracy of each indicator. For the weighted comprehensive indicator, a too-low noise-to-signal ratio will lead to a sharp increase in the weight, which in turn will seriously affect the forecasting accuracy. In contrast, the weighted average comprehensive indicator puts more weight on the signals issued by indicators and avoids the problem of excessive weight. Therefore, it is reasonable that comprehensive indicator IV performs better at both correctly calling housing price crises and at predicting housing price crises given no signal.

RETRACTED

In summary, the in-sample results from Tianjin suggest that the four comprehensive indicators are informative for predicting housing price crises. Specifically, comprehensive indicator IV performs best comprehensively considering all of the criteria.

The out-of-sample results from Tianjin reflect the out-of-sample forecasting accuracy of the four comprehensive indicators. First, the *QPS* values and noise-to-signal ratios of the four comprehensive indicators are less than 1, indicating that these indicators are useful tools for predicting housing price crises. Second, comprehensive indicator IV performs better than both comprehensive indicators I and III in terms of its ability to correctly call housing price crises. Third, comprehensive indicator IV performs better than both comprehensive indicators I and II in terms of its ability to predict non-housing price crises and to predict housing price crises given a signal. Finally, comprehensive indicator IV performs better than both comprehensive indicators I and III in terms of its ability to predict housing price crises given no signal.

Fig 4 plots the forecasted probabilities of housing price crises for the four comprehensive indicators (*k* = 1). It is obvious that some comprehensive indicators have captured the abnormal situation before a crisis. First, comprehensive indicators I, II and IV significantly exceed the cut-off probability at the end of 2016 and 2017, thus accurately predicting the occurrence of housing price crises. Second, comprehensive indicator III exceeds the cut-off probability at the end of 2016, and predicts the housing price crisis that occurred in 2016.

**Fig 4:** Probability forecasts of housing price crises for Tianjin. The shaded regions represent the time spans of housing price crises. The solid lines are the forecasted probabilities from the four comprehensive indicators with the threshold level of *k* = 1. Correspondingly, the dashed lines are their cut-off probabilities.

RETRACTED

Table 8 shows the in-sample and out-of-sample forecasting results of the four comprehensive indicators in the early warning system for Chongqing’s housing price crises.

**Table 8:** Predictive ability from the comprehensive indicators.

**In-sample** 2005Q3-2014Q2	**Chongqing**			
Comprehensive indicator	I	II	III	IV
Cut-off probability	0.45	0.35	0.45	0.35
Quadratic Probability Score	0.22	0.25	0.25	0.22
Noise-to-signal ratio	0.00	0.07	0.00	0.00
Probability of crises correctly called	0.58	0.58	0.58	0.58
Probability of safety correctly predicted	1.00	0.96	1.00	1.00
Conditional probability of crises given a signal	1.00	0.88	1.00	1.00
Conditional probability of crises given no signal	0.17	0.18	0.17	0.17
**Out-of-sample** 2014Q3-2018Q4 Quadratic Probability Score	0.60	0.57	0.65	0.51
Noise-to-signal ratio	0.00	0.33	NaN	0.00
Probability of crises correctly called	0.20	0.50	0.00	0.20
Probability of safety correctly predicted	1.00	0.83	1.00	1.00
Conditional probability of crises given a signal	1.00	0.71	NaN	1.00
Conditional probability of crises given no signal	0.40	0.33	0.45	0.40

Note: The cut-off probability for each comprehensive indicator comes from the in-sample estimation by minimizing the noise-to-signal ratio. The probability of crises correctly called is defined as *A/*(*A* + *C*); the probability of safety correctly predicted is defined as *D/*(*B* + *D*); the conditional probability of crises given a signal is defined as *A/*(*A* + *B*); the conditional probability of crises given no signal is defined as *C/*(*C* + *D*). “NaN”, standing for not a number, is a numeric data type value representing an undefined or unrepresentable value.

The in-sample results from Chongqing are interesting. First, the *QPS* values and noise-to-signal ratios of the four comprehensive indicators are less than 1, indicating that these indicators are useful tools for predicting housing price crises. Second, comprehensive indicators I, III and IV have the same performance in terms of their ability to correctly call housing price crises, to correctly predict non-housing price crises, to predict housing price crises given a signal, and to predict housing price crises given no signal. In contrast, comprehensive indicator II performs poorly across all of the criteria considered. One explanation for this result is that while the extreme comprehensive indicator contains aggregate information, it does not account for the different forecasting accuracy of each individual indicator. The weighted average comprehensive indicator puts more weight on the signals issued by indicators and avoids the problem of excessive weight. Therefore, it is reasonable that comprehensive indicator IV performs better or equal to the other comprehensive indicators across all the criteria considered.

RETRACTED

In summary, the in-sample results from Chongqing suggest that the four comprehensive indicators are informative for predicting housing price crises. Specifically, comprehensive indicators IV has a better performance than comprehensive indicator II does across all of the criteria considered.

The out-of-sample results from Chongqing reflect the out-of-sample forecasting accuracy of the four comprehensive indicators. First, the *QPS* values and noise-to-signal ratios of the three comprehensive indicators other than the weighted comprehensive indicator are less than 1, indicating that these indicators are useful tools for predicting housing price crises. It is not easy to evaluate the predictive ability of the weighted comprehensive indicator. Second, comprehensive indicator IV performs better than or equal to both comprehensive indicators I and III in terms of its ability to correctly call housing price crises. Third, comprehensive indicator IV performs better than or equal to the other three comprehensive indicators in terms of its ability to correctly predict non-housing price crises and to predict housing price crises given a signal. Finally, comprehensive indicator IV performs better than or equal to comprehensive indicators I and III in terms of its ability to predict housing price crises given no signal.

Fig 5 plots the forecasted probabilities of housing price crises for the four comprehensive indicators (*k* = 1). It is obvious that some comprehensive indicators have captured the abnormal situation before a crisis. First, comprehensive indicator I rises to the cut-off probability in 2017, and weakly predicts the price crisis that occurred in 2017. Then it rises rapidly and breaks through the cut-off probability, accurately predicting the housing price crisis that occurred in 2018. Second, comprehensive indicator II rises rapidly and significantly breaks through the cut-off probability in 2017 and 2018, accurately predicting the housing price crises that occurred in those years. Third, comprehensive indicator III remains at a stable level after 2015, and rises to the cut-off probability in 2018, weakly predicting the price crisis that occurred in 2018. Finally, comprehensive indicator IV rises linearly at the end of 2016, and breaks through the cut-off probability in 2018, thus accurately predicting the housing price crisis that occurred in 2018.

**Fig 5:** Probability forecasts of housing price crises for Chongqing. The shaded regions represent the time spans of housing price crises. The solid lines are the forecasted probabilities from the four comprehensive indicators with the threshold level of k = 1. Correspondingly, the dashed lines are their cut-off probabilities.

RETRACTED

## 4. Conclusion

In this paper, we use the KLR method to monitor a number of economic indicators that tend to exhibit abnormal behavior in the periods before a housing price crisis. On the basis of our 13 individual indicators from four major cities in China, we construct four comprehensive indicators, namely, the summed comprehensive indicator, the extreme comprehensive indicator, the weighted comprehensive indicator, and the weighted average comprehensive indicator. We also calculate the conditional probabilities of crises given a signal of the four comprehensive indicators and their cut-off probabilities. In the out-of-sample prediction, the possibility of the housing price crisis in the four cities varies with the four indicators, which also proves that the warning information reflected by different indicators is not completely the same. In particular, indicator IV constructed in this paper overcomes the problem of low accuracy in the case of low noise signal ratio.

We evaluate the in-sample and out-of-sample performance of the four comprehensive indicators for predicting housing price crises. For the four major cities in China, the in-sample forecasting results suggest that the four comprehensive indicators can be useful tools for predicting housing price crises. Specifically, the weighted average comprehensive indicator outperforms the others in terms of overall performance across all of the criteria. The out-of-sample forecasting results suggest that the weighted average comprehensive indicator performs better than the summed comprehensive indicator and the extreme comprehensive indicator in terms of overall performance across all of the criteria, making it a good comprehensive indicator to construct an early warning system for predicting housing price crises.

It should be emphasized that using a signal extraction approach, we do not establish a perfect early warning system of housing price crises. In future research, we would like to add more individual indicators to the early warning system, such as real estate loan, money-market rate, and other indicators that capture aberrant behavior in urban housing markets. In addition, it is possible to construct a new comprehensive indicator in the future, which outperforms the above four comprehensive indicators. We continue to explore these and other improvements to our early warning system. Besides, the regional policies differ from big cities and small cities, constructing the emergency system of small city is also a valuable theme that could be taken into consideration.
